The article "Comprehensive Evaluation of College Students' Physical Health and Sports Mode Recommendation Model Based on Decision Tree Classification Model" was published in 2022. Journal: Comput Intell Neurosci.

# Comprehensive Evaluation of College Students' Physical Health and Sports Mode Recommendation Model Based on Decision Tree Classification Model

**DOI:** 10.1155/2022/5504850

**Published:** 2022-07-22

**Authors:** Wenzheng Chen, Guanglei Yang, Dongkai Qi

**Affiliations:** ^1^Basic Teaching Department, Chengdu Aeronautic Polytechnic, Chengdu, Sichuan 610100, China; ^2^Department of Computer Science, College of Computing, Illinois Institute of Technology, Chicago, IL 60616, USA

## Abstract

Nowadays, more and more college students' physical health is getting worse because of their living habits and self-consciousness. In order to improve the physical quality of college students as much as possible, the experiment uses the improved iterative dichotomiser III (ID3) decision tree to make decisions on the physical condition of some college students and the corresponding sports mode recommendation, and compares the results with the traditional ID3 algorithm. In the experimental results, the information entropy ratio of the improved ID3 algorithm is 89.5%, the operation information loss rate is 4.136%, and the accuracy of motion mode decision is 92.58%. The average relative time is 12.7, and the accuracy of physical health decision making is 90.02%. The above two values are not significant compared with the traditional ID3 algorithm. The experimental results show that the improved ID3 algorithm has significant optimization in the stability of information transmission and the accuracy of sports recommendation decision making, and can be applied to the physical health evaluation and sports recommendation of college students in a certain range.

## 1. Introduction

College students are backbones of society. It is particularly important for college students to maintain their physical health. However, with the development of society, more and more college students have health problems [1]. Many college students' health conditions gradually deteriorate due to bad living habits, and their cardiopulmonary function, muscle strength, and flexibility are difficult to meet the standard [2]. In addition, some college students do not pay enough attention to their own physical health, and some colleges and universities themselves lack attention to the health of college students. They do not recommend appropriate sports modes for students' possible physical health [3]. Some studies in recent years have also found that the physical health level of college students has decreased significantly compared with previous years [4].

In view of the above situations and problems, the experiment uses an improved ID3 algorithm to construct the decision tree and gives the corresponding physical health indicators and recommended exercise patterns for college students according to the decision results. ID3 algorithm takes the initial set as the root node. In each iteration of the algorithm, it traverses each attribute in the set and calculates the entropy or information gain of the attribute. We select the attribute with minimum entropy or maximum information gain. Then, the selected attributes are used to divide the set into different data subsets. The algorithm continues to recursively process each subset, and only the previously unselected attributes are considered each time. In the recursive process of subset, if each element in the subset belongs to the same class, or there are no more attributes to choose from in the subset, or there are no instances in the subset, the recursion will end. In the whole algorithm, the branch node in the decision tree represents the selected data of the segmented data, and the terminal node represents the class label of the final subset of this branch. The improvement of ID3 is to construct a new attribute and multivariable decision tree and generate it in the form of binary tree to increase the accuracy and operation speed.

The article "Comprehensive Evaluation of College Students' Physical Health and Sports Mode Recommendation Model Based on Decision Tree Classification Model" was published in 2022. Journal: Comput Intell Neurosci.

The innovation of this paper is to design an improved ID3 according to the defects of ID3 and compare the improved ID3 with the traditional ID3. In addition to the decision accuracy, the compared test data also include the operation rate and the parameters related to the stability of information transmission, so as to obtain a more objective experimental conclusion. The experimental results show that the improved ID3 algorithm is better than the traditional ID3 algorithm in terms of operation speed, information entropy reduction, health decision accuracy, sports mode recommendation accuracy, and operation information loss rate. However, only the information entropy is reduced, and there is a significant difference between the accuracy of motion mode recommendation and the loss rate of operation information, indicating that the improved ID3 has significantly improved the stability of data transmission, and the improvement of accuracy and operation speed is not significant, respectively.

The article is mainly divided into four parts. The first part mainly expounds the experimental research background and significance of the article in detail, describes the research methods and innovations in more detail, and introduces the article structure. The second part mainly describes the generation of ID3 algorithm decision tree, the improvement method designed according to the shortcomings of traditional ID3, and the construction of evaluation system. The third part mainly explores the experimental results of each index between the improved ID3 algorithm and the traditional ID3, compares, and analyzes the experimental results, and the fourth part is the experimental conclusion based on the experimental results and analysis, and puts forward the shortcomings of the research and the prospect of future research.

The article "Comprehensive Evaluation of College Students' Physical Health and Sports Mode Recommendation Model Based on Decision Tree Classification Model" was published in 2022. Journal: Comput Intell Neurosci.

## 2. Related Work

At present, many scholars at home and abroad have studied decision tree classification such as ID3. Meng and Wang proposed a new ID3 decision tree model and applied it to English learning. Through ID3 to classify English semantics, the experimental results show that the accuracy is 63.6%, which is higher than the previous decision tree model [5]. Haidar et al. synthesized C4 5 algorithm and ID3 algorithm, select multiple index sample data, and use it to predict students' DROPOUT according to the decision results. The results show that the accuracy rate is as high as 94.7% [6]. Rosid et al. used the improved ID3 algorithm to classify dengue hemorrhagic fever and strengthened the prevention and treatment of the disease according to the classification results. The experimental results showed that the classification accuracy reached 82% [7]. Koren et al. used C4 5. ID3, k-nearest neighbor algorithm, has been combined with radial basis function and other decision trees to classify various characteristics of 21 kinds of beer in detail and evaluate relevant factors, and finally design the function of flavonoid content, glucose, fructose, sucrose, and other factors with color and bitterness [8]. In order to protect privacy data mining, Li et al. used ID3 algorithm to make decision protection for cloud data transmission, which not only improved the protection performance of privacy but also reduced the cost [9]. After comprehensively comparing different types of decision trees, Maingi et al. adopted the improved ID3 algorithm to jointly monitor the spread of possible diseases in different geographical regions and prevent disease outbreaks. Finally, it achieved certain results in disease prevention and control [10].

Vasquez and Comendador used ID3 algorithm to judge the working technology and learning ability that high school students have mastered at present, and make recommendation decisions for students, so as to judge the suitable direction of students' study in the future university [11]. Pang collected the evaluation data set of teaching assistants from the university machine learning database, established ID3 decision tree based on these data, and found the maximum information gain in different iteration levels. The final results showed that the decision tree effectively evaluated the work progress of 151 teaching assistants and improved their work ability [12]. In order to accelerate the development of the sports and fitness industry, Gu and He used ID3 fuzzy decision tree to build a tree according to the characteristics of customer data and the loss of customers, and analyzed the main factors of customer changes. Finally, it was concluded that the accuracy of ID3 fuzzy decision tree was as high as 97.8%, which could accurately analyze the causes of customer loss [13]. Li et al. have designed a system based on ID3 and C4 5. The new decision algorithm is applied to the performance evaluation and analysis of new energy vehicles, and the accuracy and time complexity between the new decision tree and the traditional algorithm are compared. The results show that the new decision algorithm has higher accuracy and lower time complexity [14]. Mebawondu et al. comprehensively used a variety of decision tree algorithms; fully applied modern digital technology to the agricultural department to monitor physical, biological, and microbial changes; and accurately classified the types and quality of raw materials. The final experimental results showed that the accuracy of the research reached 98.75%, which can be applied to the monitoring of the agricultural department.

The article "Comprehensive Evaluation of College Students' Physical Health and Sports Mode Recommendation Model Based on Decision Tree Classification Model" was published in 2022. Journal: Comput Intell Neurosci.

From the above research, it can be seen that ID3 decision tree is widely used and can play its role in many fields. There are more research types on students' decision making, while there are relatively few decisions for college students' physical health. The experiment uses the traditional ID3 algorithm and the improved ID3 algorithm to compare, hoping to get a more effective decision tree algorithm, so as to apply it to the decision making of college students' physical health.

## 3. Application of ID3 Algorithm and Its Improved Algorithm in College Students' Physical Health Decision Making

### 3.1. Construction of ID3 Algorithm Decision Tree and Its Improved Algorithm

ID3 algorithm is the most commonly used algorithm in building decision tree model. It has certain solutions, strong learning ability, comprehensive use of training data, continuous processing of discrete fields, and generation of understandable rules, and the amount of calculation will not be too large. This algorithm is suitable for dealing with large-scale learning problems. Its process is divided into main algorithm and ID3 tree building algorithm [15]. The main algorithm needs to randomly select a subset containing both positive and negative examples from the training sample set as the window and use ID3 algorithm to randomly generate a decision tree for the above subset. Its basic process is shown in Figure 1 [16]. Where TE1 and TE2 are subsets of the positive example set te, and Fe1 and Fe2 are subsets of the negative example set Fe.

The article "Comprehensive Evaluation of College Students' Physical Health and Sports Mode Recommendation Model Based on Decision Tree Classification Model" was published in 2022. Journal: Comput Intell Neurosci.

The construction of decision tree model is based on information entropy. In information transmission, the information transmitted in the source includes a limited number of mutually exclusive and joint complete times. The average of the probability of these times is the information entropy. Similar to the meaning of entropy in thermodynamics, information entropy is also a statistic expressing the degree of chaos of information system. The lower the value of information entropy, the more orderly the construction of information system [17]. Therefore, the construction of decision tree should minimize the amount of information entropy. When ID3 builds a tree, each nonleaf node in the decision tree corresponds to a noncategory attribute, the branch is the value of the attribute, and a leaf node represents the value of the category attribute corresponding to the path from the tree root to the leaf node. Then, each nonleaf node will be associated with the noncategory attribute with the largest amount of information in the attribute. Finally, information gain is used to select the attributes that can best classify the samples [18].

ID3 algorithm selects the attribute with the highest information gain as the test attribute of the current node, which minimizes the information required for sample classification of result division and reflects the lowest randomness of division [19]. Let *S* be a collection of *s* result data samples, and the class label attribute has *n* different values and *n* different *C*_*i*_, (*i* = 1, 2, 3,…, *n*). Let *S*_*i*_ be the number of samples in class *C*_*i*_, and the expected information required for the classification of a given sample is shown in equation (1). In formula (1), *p*_*i*_ represents the probability that any sample belongs to *C*_*i*_.

(1) $$\begin{array}{c} I\left(s_{1},s_{2},\ldots ,s_{n}\right)=-\sum_{i=1}^{n}p_{i}\log_{2}\left(p_{i}\right). \end{array}$$

An attribute *A* can have a different value range {*a*_1_, *a*_2_,…, *a*_*r*_}. Through the attribute *A*, the set *S* can be divided into *r* different subsets {*s*_1_, *s*_2_,…, *s*_*r*_}. *S*_*i*_ contains the corresponding data sample *a*_d_ that is the d value in the attribute *A* of the set *S*. If attribute *A* is the test attribute and *S*_*i*d_ is the number of samples belonging to category *C*_*i*_ in the subset *S*_d_, the required information for analyzing the current sample set according to attribute *A* is as follows:

(2) $$\begin{array}{c} E\left(A\right)=\sum_{d=1}^{r}\frac{s_{1d}+s_{2d}+\cdots +s_{md}}{s}I\left(s_{1d},s_{2d},\ldots ,s_{md}\right). \end{array}$$

In equation (2), *s*_1*d*_+*s*_2*d*_+⋯+*s*_*md*_/*s* term is used as the weight of the *d* subset. The smaller the value of *E*(*A*), the better the subset division. For a given subset *S*_*d*_, the information is as follows (3). In equation (3), *p*_*id*_ is the probability of any data sample in subset *S*_*d*_.

(3) $$\begin{array}{c} I=-\sum_{i=1}^{n}p_{id}\log_{2}\left(p_{id}\right). \end{array}$$

At this time, the information income *G*(*A*) can be obtained, as shown in formula (4). Information gain *G*(*A*) is the reduction of information entropy. Therefore, the greater the value, the higher the degree of regularity of system information.

(4) $$\begin{array}{c} G\left(A\right)=I-E\left(A\right). \end{array}$$

ID3 algorithm also has some shortcomings and problems. The algorithm may converge locally, resulting in the loss of optimal solution. The continuous algorithm is difficult to predict. When there are too many categories, it is prone to many errors, the amount of calculation is too large, and it may not be able to accurately select the best attribute [20]. Therefore, in order to make ID3 algorithm achieve its optimal effect, the algorithm must be improved accordingly.

The article "Comprehensive Evaluation of College Students' Physical Health and Sports Mode Recommendation Model Based on Decision Tree Classification Model" was published in 2022. Journal: Comput Intell Neurosci.

Aiming at the problem of attribute interaction and subtree repetition, the method of modifying the test attribute space is mainly adopted. This method is mainly based on data-driven construction, combining some attributes through mathematical or logical operators to construct new attributes and new multivariable decision tree, or based on hypothesis driven construction, using simple logical operators to construct new attributes to change attribute space and learning mode, and then establishing a new decision tree on the new attribute space and executing recursively until the end [21]. Therefore, the core idea of the improvement of ID3 algorithm is to reduce the information entropy in ID3 algorithm to improve the tree building speed and efficiency, and change the data structure so that its value is no longer biased toward the attribute with the most values, but toward the optimal solution. Let the training instance set be *X*, the total number of training instances in *X* is |*X*|, and the number of training instances of class *i* is |*X*_*i*_|. The probability that an instance belongs to class *i* is *P*(*X*_*i*_). The information entropy *H*(*X*) at this time can be obtained, as shown in the following equation.

(5) $$\begin{array}{c} H\left(X\right)=-\sum_{i=1}^{n}P\left(X_{i}\right)\log_{2}P\left(X_{i}\right). \end{array}$$

At this time, a decision tree can make correct category judgment for a single instance, and the amount of information required is shown in equation (6). In equation (6), *S* is the original set, *P* is the probability, and *N* is the number of attributes.

(6) $$\begin{array}{c} E\left(S\right)=-\frac{P}{N+P}\log\frac{P}{N+P}-\frac{N}{N+P}\log\frac{N}{N+P}. \end{array}$$

The decision tree represents the conjunctive disjunction of instance attribute value constraints. Each path from leaves to tree roots corresponds to the conjunction of a set of attribute tests, and the tree itself corresponds to the disjunction of this conjunction. Since the learning of decision tree is the process of reducing the uncertainty of decision tree division and increasing the stability of information, when testing attribute *F*, let it be attribute value *f*_1_, *f*_2_,…, *f*_*n*_. If *F* = the value *f*_*j*_ of item *j*, the number of instances of class *i* is |*X*_*ij*_|, and the probability of belonging to class *i* is *P*(*X*_*i*_*|F*=*f*_*j*_). We record the instance set of *F*=*f*_*j*_ as *Y*_*j*_, and equation (7) is obtained at this time.

(7) $$\begin{array}{c} H\left(Y_{j}\right)=-\sum_{i=1}^{n}P\left(X_{i}|F=f_{j}\right)\log_{2}P\left(X_{i}|F=f_{j}\right). \end{array}$$

The information entropy of each subset recorded by node *F* according to test attribute *F* is recorded as *H*(*X|F*). According to the principle of information entropy and equivalent substitution, equations (8) and (9) are obtained, respectively.

(8) $$\begin{array}{c} H\left(X|F\right)=\sum_{j=1}^{t}\sum_{i=1}^{n}P\left(F=f\right)P\left(X_{i}|F=f_{j}\right)\log_{2}P\left(X_{i}|F=f_{j}\right), \end{array}$$

(9) $$\begin{array}{c} E\left(X_{i}\right)=-\sum_{j=1}^{n}\frac{P_{ij}}{\left|X_{i}\right|}\log\frac{P_{ij}}{\left|X_{i}\right|}. \end{array}$$

Let the number of positive case sets be *p*, and the number of negative case sets be *n*. When *F*=*f*_*j*_, the branch has *p*_*i*_ positive case sets and *n*_*i*_ negative case sets. Because the information gain value *G*(*F*) is the reduced value of information entropy, the final simplified information gain value *G*`(*F*) is obtained from McLaughlin formula when *x*⟶0, ln(1+*x*) ≈ *x* − 1/2*x*^2^, as shown in the following equation.

(10) $$\begin{array}{c} G`\left(F\right)=\sum_{j=1}^{t}\frac{p_{j}n_{j}}{p_{j}+n_{j}}. \end{array}$$

Combining the simplified algorithm with binary tree, the binary tree gain algorithm of ID3 simplified algorithm is obtained. The basic principle of the improvement is to consider the attributes and attribute values in the binary tree, avoid the disadvantage of only taking attribute classification, and take into account the proportion of information gain and attribute value. Since there are only two final values of each attribute (*Y* or *n*), the decision tree formed is a binary tree [22]. The simplified diagram of the newly generated tree is shown in Figure 2. Binary tree can iterate the input data layer by layer to get different decision classifications. It not only reduces the information entropy and speeds up the operation speed, but also has many kinds of decision results.

The article "Comprehensive Evaluation of College Students' Physical Health and Sports Mode Recommendation Model Based on Decision Tree Classification Model" was published in 2022. Journal: Comput Intell Neurosci.

### 3.2. Construction of College Students' Physical Health Evaluation System and Application of Improved ID3 Algorithm

Because there are many kinds of indicators that can evaluate the physical health of college students, each has its own importance. Therefore, in order to get an accurate and comprehensive evaluation, the construction of the evaluation system needs to meet the principles of scientificity, independence, goal consistency, guidance, and operability. On the basis of these principles, the experiment adopts the interactive hierarchical structure, there is a subordinate relationship between each layer, and at the same time, the secondary indicators intersect with each other, and the index map of college students' physical fitness evaluation is formulated by integrating the standards of college students' physical examination. The physical test indexes of college students include BMI, vital capacity, sitting forward flexion, standing long jump, running 50 m, 1000 m male/800 m female, and pull-up male/1-minute sit-up female plus vision test (no score). This paper only shows some evaluation results, as shown in Figure 3.

For each secondary index, the experiment uses analytic hierarchy process (AHP) to determine the relevant weight of each index. AHP is a method that hierarchizes the problem, compares each index at the same level, judges the importance, and obtains the weight [23]. When using AHP, we should first clarify the scope, structure, and content of the evaluation index and then establish a hierarchical structure according to the hierarchy and subordinate relationship. The highest level represents the goal of the problem and usually has only one element, the middle is the criterion level, and the lowest level is the measure level, which will be constrained by the elements of the upper level. Then, the judgment matrix is constructed to judge the relative importance of each index according to the scaling method. In the scaling method, the corresponding scaling value will be obtained according to the relative importance between the two elements, so as to quantify the judgment results and construct the judgment matrix, as shown in the following equation:

(11) $$\begin{array}{c} M=\left[\begin{array}{cccc} m_{11}, & m_{12}, & \ldots , & m_{1n}\\ m_{21}, & m_{22}, & \ldots , & m_{2n}\\ \ldots \\ m_{n1}, & m_{n2}, & \ldots , & m_{nn} \end{array}\right]. \end{array}$$

The matrices in equation (11) satisfy *m*_*ii*_=1 and *m*_*ij*_=*m*_*ji*_ because of the symmetry principle. Then, we calculate the weight, normalize the judgment matrix, and divide it by the sum of each column to make them sum to 1, as shown in the following equation:

(12) $$\begin{array}{c} t_{ij}=\frac{m_{ij}}{\sum_{j=1}^{n}t_{ij}},T=\left[t_{ij}\right]. \end{array}$$

We sum each row of the normalized matrix and then calculate the eigenvector of the matrix, which is the weight vector, as shown in equation (13). In equation (13), the sum value of each row is as follows:

(13) $$\begin{array}{c} w_{i}=\frac{v_{i}}{\sum_{i=1}^{n}v_{i}},\\ W=\left[w_{i}\right]. \end{array}$$

Finally, the consistency of the judgment matrix is tested. For the maximum eigenvalue *λ*_max_ of the order judgment matrix, if *λ*_max_=*n*, it has complete consistency. Otherwise, the consistency ratio needs to be calculated, as shown in the following equation:

(14) $$\begin{array}{c} \text{CR}=\frac{\text{CI}}{\text{RI}}. \end{array}$$

In equation (14), CR is the consistency ratio, RI is the average random consistency index value, and CI is the consistency index. The calculation of consistency index is shown in equation (15). In equation (15), AW is the product of judgment matrix and eigenvector. When the result of CR is less than 0.1, it is considered that the result of the judgment matrix is consistent and passes the consistency test.

(15) $$\begin{array}{c} \left\{\begin{array}{c} \text{CI}=\frac{\lambda_{\max}-n}{n-1},\\ \lambda_{\max}=\frac{1}{n}\sum_{i=1}^{n}\frac{{\left(AW\right)}_{i}}{w_{i}}. \end{array}\right. \end{array}$$

The value of RI according to its order is shown in Figure 4. According to the above method, the CR value in the experiment is 0.069 < 0.1, so it passes the consistency test.

The article "Comprehensive Evaluation of College Students' Physical Health and Sports Mode Recommendation Model Based on Decision Tree Classification Model" was published in 2022. Journal: Comput Intell Neurosci.

Figure 4 shows the RI measurement diagram with orders. After completing the above steps, the experiment carries out the evaluation system setting, index weight setting, comprehensive evaluation calculation, and decision tree analysis of the computer system according to the indexes and weights. The experiment uses the improved ID3 in the analysis of computer system decision tree, compares the improved ID3 algorithm with the unmodified ID3, and selects some sample data for operation decision classification. 300 college students were randomly divided into 5 groups with 30 college students in each group [24]. After testing their indicators, 150 of them were randomly selected as the training set, and the remaining data were collected as the test set and preprocessed. The preprocessing method is to clean up the data first. For incomplete data, you can ignore tuples and use attribute average value; then, it is data reduction, which deletes attributes that are not related to data mining or have a low degree of correlation. Finally, the data are discretized. According to the score of each secondary index of students, it is divided into four levels: 85–100 is excellent, 75–85 is good, 60–75 is medium, and less than 60 is poor. The decision tree will classify the primary indicators according to the decision results of the secondary indicators and then make the overall decision according to the results of the primary indicators [25].

## 4. Analysis of Decision Results of ID3 Algorithm and Its Improved Algorithm

The experiment uses a scoring system. Each student scores the decision results obtained from the two decision trees according to their satisfaction, with a full score of 100. The traditional ID3 decision tree and the improved ID3 decision tree are used to calculate and obtain the decision results. The average operation rate and operation information loss rate were calculated for each group. In addition to the operation speed and the loss rate of operation information, the accuracy of decision making is equally important, but it is difficult to directly quantify the accuracy of decision making. Therefore, the experiment calculates the information entropy ratio at the same time and calculates the information entropy ratio of each group of data of improved ID3 and traditional ID3, in order to compare the accuracy and stability of information transmission. Because each student scores the two algorithms at the same time, the average value of the score can reflect the classification results of the decision tree and the accuracy of the recommended motion patterns according to the results to a certain extent, so the average result is taken as the accuracy. Although the subjective criteria and strictness of each student's score are different, the decision tree will recommend the corresponding exercise mode according to the decision results of the primary and secondary indicators.

The experiment uses two methods to generate decisions for the five groups of data randomly grouped, and their respective relative operation time is shown in Figure 5. It can be seen from Figure 5 that the relative operation time of the improved ID3 in the five groups of experiments is the shortest. Compared with the traditional ID3, the time ratios of each group are 0.95, 0.91, 0.97, 0.93, and 0.96, respectively. From the average results, the average relative time of the improved ID3 is 12.7, the average relative time of the traditional ID3 is 13.5, and the average time ratio is 0.94, indicating that the operation speed of the improved ID3 has been improved, but the time ratio is mostly about 0.95, so the improvement is not significant enough.

The article "Comprehensive Evaluation of College Students' Physical Health and Sports Mode Recommendation Model Based on Decision Tree Classification Model" was published in 2022. Journal: Comput Intell Neurosci.

The information entropy ratio of each group of experiments is shown in Figure 6. As can be seen from Figure 6, the results of each group of experimental data are less than 100%, indicating that the number of information entropy of the improved ID3 algorithm is reduced to a certain extent compared with the traditional ID3 algorithm. From the average value, the lowest information entropy ratio is 86.55%, indicating that the information entropy contained in the improved ID3 is less than 90% of the traditional ID3, which is significant. The variation range between each group of data is also small, and the variance of all data is 2.56, indicating that the stability of the improved ID3 decision-making operation process is high.

We feed back the results of the decision tree to the corresponding college students and collect their scoring data. The average score of each group for physical health decision making is shown in Figure 7. It can be seen from Figure 7 that the average score of the improved ID3 algorithm is higher in the results of each group except group 4, but the gap between the five groups of data is not significant. The ratios of the score of the improved ID3 algorithm and the ID3 result of each group of data are 1.0096, 1.0098, 1.0014, 0.996, and 1.0128, respectively. Except group 5, the absolute value of the difference between each group of data and 1 is less than 0.01, which shows that the gap value is very small. It is impossible to intuitively decide whether ID3 can be improved. Taking the score as the accuracy reference, the accuracy of improved ID3 is 90.02%, and that of traditional ID3 is 89.49%.

ID3 decision tree will recommend the corresponding sports types and patterns for each college student according to the decision classification results of the indicators. The average results of each college student's scoring according to their recommendation decisions are shown in Figure 8. It can be seen from Figure 8 that the average score of each group of data is higher than that of the traditional ID3 algorithm, and it can be seen intuitively that the higher score is more significant. Among them, the score ratios of each group were 1.056, 1.066, 1.035, 1.047, and 1.026, respectively, which were greater than 1.01. Therefore, it can be seen that the improved ID3 algorithm is more accurate than the traditional ID3 algorithm in the decision making of motion mode recommendation. Taking the score as the accuracy reference, the accuracy of the improved ID3 is equivalent to the sum of the average scores of each group, and then, we take the percentage, that is, 92.58%, which is significantly higher than 88.49% of the traditional ID3.

The article "Comprehensive Evaluation of College Students' Physical Health and Sports Mode Recommendation Model Based on Decision Tree Classification Model" was published in 2022. Journal: Comput Intell Neurosci.

The information loss rate calculated by the two algorithms is shown in Figure 9. As can be seen from Figure 9, except the first group, the data of other groups are improved ID3, the information loss rate is lower than that of traditional ID3, and the results of the remaining four groups are significantly different. In order to further compare the difference in the operation information loss rate between the two and calculate the average value of each group of results, the operation information loss rate of the improved ID3 is 4.136%, while the operation information loss rate of the traditional ID3 is 4.508%. Therefore, it can be concluded that the operation information loss rate of the improved ID3 algorithm is significantly lower than that of the traditional ID3 algorithm and is more stable in information transmission.

## 5. Conclusion

This paper uses the improved ID3 decision tree to make decisions on various indicators of college students' health, and makes sports mode recommendation decisions according to the results, and compares it with the traditional ID3 algorithm. The improved ID3 algorithm is superior to the traditional ID3 algorithm in terms of operation speed, information entropy reduction, health decision accuracy, sports mode recommendation accuracy, and operation information loss rate. However, it only reduces the information entropy, and there is a significant difference between the accuracy of motion mode recommendation and the loss rate of operation information. It shows that the improved ID3 has significantly improved the stability of data transmission. The improvement of accuracy and operation speed is not significant, respectively. Although the research has achieved some results, the number of samples is relatively small, the accuracy of the test method is the scoring system, and the degree of rigor is not high enough. In the follow-up research, it is necessary to further select more and more representative sample data and design a better accuracy test scheme, which is also a problem that needs to be improved in further research in the future.

## Figures and Tables

**Figure 1:** Simple flowchart of ID3 main algorithm.

**Figure 2:** Simplified diagram of binary tree gain algorithm.

**Figure 3:** Physical health evaluation index.

**Figure 4:** Metering diagram of RI with order.

**Figure 5:** Relative time diagram of two algorithms.

**Figure 6:** Information entropy ratio diagram.

**Figure 7:** Scoring chart for physical health results.

**Figure 8:** Scoring chart for sports mode recommendation.

The article "Comprehensive Evaluation of College Students' Physical Health and Sports Mode Recommendation Model Based on Decision Tree Classification Model" was published in 2022. Journal: Comput Intell Neurosci.

**Figure 9:** Statistical chart of operation information loss rate of two algorithms.

## Data Availability

The data used to support the findings of this study are included within the article.
